The article "Prevalence of complications among Chinese diabetic patients in urban primary care clinics: a cross-sectional study" was retracted in 2025. Reason: lack of ethics approval or compliance.

# Prevalence of complications among Chinese diabetic patients in urban primary care clinics: a cross-sectional study

**DOI:** 10.1186/1471-2296-15-8

**Published:** 2014-01-10

**Authors:** Kenny Kung, Kai Ming Chow, Eric Ming-Tung Hui, Maria Leung, Shuk Yun Leung, Cheuk Chun Szeto, Augustine Lam, Philip Kam-Tao Li

**Affiliations:** 1 Department of Family Medicine, New Territories East Cluster, Hospital Authority, Shatin, Hong Kong; 2 Department of Medicine and Therapeutics, Prince of Wales Hospital, Chinese University of Hong Kong, 32, Ngan Shing Street, Shatin, Hong Kong

**Keywords:** Diabetic complications, Primary care, Chronic illness, Screening program

## Abstract

**Background:**

A territory-wide diabetes management program (Risk Assessment Management Program – RAMP) was recently established, providing comprehensive management for all diabetics, helping to delineate current level of control and complications prevalence among primary care diabetic patients in Hong Kong.

**Method:**

This cross-sectional study captured anonymous clinical data from RAMP patients. Data obtained include sociodemographic details, type of diabetes, illness duration, family history, drug usage, coexisting illnesses, diabetic complications and other clinical parameters.

**Results:**

Data from 15,856 type 2 diabetic patients were analyzed. 57.1% were above 60 years old, with mean disease duration of 7.3 years. Hypertension was the commonest coexisting chronic illness (57.6%). 30.2% and 61.8% have their systolic and diastolic pressure controlled to below 130 mmHg and 80 mmHg respectively. Over half (51.5%) had an HbA1c level of less than 7.0%. 88.4% did not achieve target lipid level. 15% were on diet control alone. Only 22.2% were on statins. In patients with microalbuminuria and macroalbuminuria, 40.7% and 54.5% were on angiotensin converting enzyme inhibitor (ACEI) or angiotensin receptor blocker (ARB) respectively. 12.9%, 38.8% and 2.4% had diabetic retinopathy, nephropathy and neuropathy respectively. Overall, 37.9%, 7.3% and 0.4% had single, two and three concurrent microvascular complications respectively.

**Conclusion:**

The level of diabetic control is comparable with other developed countries. We demonstrated a high prevalence of microvascular complications among Chinese primary care patients despite achieving adequate HbA1c levels, highlighting the importance of managing all aspects of diabetes including weight, lipid and blood pressure. Efforts to improve holistic management must be tailored according to the needs of our population, with the challenges that the majority have low educational background and in the older age group.

## Background

According to the latest information from the World Health Organization, around 346 million people worldwide have diabetes [1]. Although figures vary with estimation methods from different organizations [2,3], there is consensus that the prevalence of diabetes will continue to rise, increasing the burden to our limited healthcare resources.

The article "Prevalence of complications among Chinese diabetic patients in urban primary care clinics: a cross-sectional study" was retracted in 2025. Reason: lack of ethics approval or compliance.

Over the last few years, Hong Kong’s public primary care has introduced a new diabetes management service (Risk Assessment Management Program – RAMP) that provides comprehensive management for all diabetic patients, including annual blood tests, and two-yearly examination for retinopathy, neuropathy and nephropathy. All information is recorded electronically, allowing healthcare providers to review patients’ conditions in a much more effective and efficient way. This has also enabled healthcare providers to review the level of control and prevalence of complications among diabetic patients.

Previous studies looking into data in our locality have estimated prevalence using previous publications. A local reference framework for diabetes [4] was established in 2010, emphasizing the need for a comprehensive management of diabetes in the primary care setting. However, there is currently limited primary care data on the level of control and the prevalence of complications, which are essential in helping service providers to correctly allocate healthcare resources. Moreover, extrapolation from existing data may prove ineffective because of the substantial variation across different countries, which in turn is related to differences between populations and healthcare systems. Data from RAMP therefore provides an exceptional opportunity to delineate the current level of control and prevalence of complications among primary care diabetic patients in Hong Kong.

## Method

This study is a cross-sectional study, collecting anonymised computerized clinical data obtained from RAMP in eight public primary care clinics of Hong Kong. The public primary care system in Hong Kong provides service to patients with chronic illness, as well as socioeconomically deprived patients with episodic illnesses. Overall these eight clinics look after around 200,000 patients, amongst which around 20,000 have diabetes. Only data from patients’ first visit to RAMP were included. In order to be eligible for RAMP, patients must have a pre-existing diagnosis of diabetes. Information obtained in RAMP was recorded in the computerized Clinical Management System; patient data were anonymized by the computer system before they were drawn for analysis.

We obtained information including sociodemographic details, type of diabetes, duration of diabetes, family history of diabetes, compliance to treatment (patients’ self-report), drug usage (including both diabetes and non-diabetes related), presence or absence of coexisting conditions according to patient’s clinical history and past medical records (including systemic hypertension, coronary heart disease, cerebrovascular disease, heart failure, cataract, glaucoma, erectile dysfunction and claudication), presence or absence of specific clinical findings (including numbness and pinprick sensation), foot abnormalities (including graduated tuning fork test and 10 g monofilament test) and ankle jerks (performed by trained diabetes nurses). The following parameters were also retrieved: visual acuity (using Snellen chart assessment), blood pressure (measured with electronic sphygmomanometer), body weight, height, waist hip ratio, HbA1c, lipid profile, fasting glucose, eGFR (MDRD) and spot urine albumin to creatinine ratio (uACR) (all tests performed in accredited government hospitals’ laboratories). Retinal examination was performed by a trained optometrist using retinal photography. Two fields of the retina would be photographed for each eye. One photo was centred at the macula and the other at the optic disc. A quality assured grading system with ophthalmologist support was in place to ensure the retinopathy grading results were accurate. All photographs were reviewed by a trained optometrist. Another trained optometrist would act as the secondary grader for all abnormal retinal photographs and 15% of the retinal photographs reviewed as normal by the first optometrist. When there was disagreement, the ophthalmologist made the final decision.

The article "Prevalence of complications among Chinese diabetic patients in urban primary care clinics: a cross-sectional study" was retracted in 2025. Reason: lack of ethics approval or compliance.

The definitions used for specific variables are as follows:

1. Retinopathy

a. Mild non-proliferative (NPDR) – microaneurysms

a. Moderate to severe NPDR – microaneurysms and other microvascular lesions, including venous beading ≥2 quadrants, or intraretinal microvascular abnormalities ≥1 quadrant but not proliferative diabetic retinopathy

a. Proliferative – neovascularisation of optic disc or elsewhere, preretinal haemorrhage, or vitreous haemorrhage

2. Nephropathy

a. Overt – uACR >300 mg/g (or > 34 mg/mmol)

a. Incipient nephropathy – uACR 30–300 mg/g (or 3.4-34 mg/mmol)

a. Normoalbuminuria – normal uACR (<30 mg/g or <3.4 mg/mmol)

3. Neuropathy - Defined as presence of abnormal monofilament test or gradated tuning fork test

### Statistical analysis

Statistical analysis was performed by SPSS for Windows version 18.0 (SPSS Inc., Chicago, IL). All data are expressed as mean ± standard deviation unless otherwise specified.

### Ethical considerations

Application for ethics approval was initially considered before the start of the study. Nevertheless, taking into account that all data were drawn in an anonymized manner, and that data obtained for this study was part of the RAMP audit process, ethical approval from local ethics committee was finally considered unnecessary.

The article "Prevalence of complications among Chinese diabetic patients in urban primary care clinics: a cross-sectional study" was retracted in 2025. Reason: lack of ethics approval or compliance.

## Results

### Patient demography

From 1 Oct 2009 to 31 Dec 2011, 15,856 diabetic patients from the eight specified clinics have received care under RAMP. All were type 2 diabetics. Their sociodemographic details are shown in Table 1. 57.1% of the patients were above 60 years old, and 51.2% were female. The mean duration of diabetes among our patients was 7.3 years (SD 6.2). 58% of the population had education level of primary school or below.

**Table 1:** Sociodemographics of study population

**Characteristic**		
**Gender**	Female	51.2%
	Male	48.8%
**Age group**	20-29	0.1%
	30-39	1.1%
	40-49	9.2%
	50-59	32.4%
	60-69	29.4%
	70-79	20.7%
	80-89	6.8%
	>89	0.2%
**Smoking status**	Never-smoked	71.6%
	Ever-smoked	28.4%
**Alcohol intake**	Non-drinker	76.1%
	Ever-drinker	23.9%
**Education level**	None	18.0%
	Primary	40.2%
	Secondary	37.0%
	Tertiary or above	4.8%
**Occupation**	Housewife	28.8%
	Professional	1.9%
	Non-manual	10.6%
	Manual skilled	10.4%
	Manual non-skilled	8.8%
	Unemployed	4.3%
	Retired	35.2%
**Body mass index**	<18.5	1.2%
	18.5-22.9	22.3%
	23-24.9	21.9%
	25-27.4	26.3%
	27.4-30	15.8%
	>30	12.4%
Waist hip ratio*	Low (<0.8 female; <0.96 male)	25.8%
	Moderate (0.81-0.85 female; 0.96-1.0 male)	28.0%
	High (>0.85 female; >1.0 male)	46.2%
**Home monitoring**	None	62.2%
	Urine testing only	1.1%
	Finger prick testing	36.3%
**Mean duration of diabetes**		7.3 years
**Comorbidities**	Hypertension	57.6%
	Coronary heart disease	3.8%
	Stroke	4.5%

### Comorbidities, disease control and drug use

Hypertension was the commonest coexisting chronic illness in our population (57.6%), while less than 5% are known to have coronary heart disease and stroke (Table 1). The mean systolic blood pressure (SBP) and diastolic blood pressure (DBP) are 138 mmHg (SD 18.3) and 76 mmHg (SD 10.5) respectively (Table 2) with a relatively normal distribution (first and third quartile for SBP being 127 and 151 mmHg, and DBP 69 and 83 mmHg respectively). Blood pressure control (below 130/80 mmHg) was achieved in 22.9% and 35.9% of patients with and without a prior diagnosis of hypertension respectively (p < 0.001).

**Table 2:** Lipid profile and eGFR among study population

**Mean blood pressure**		
Systolic	138 mmHg	(18.3)
Diastolic	76 mmHg	(10.5)
**Mean lipid profile**		
TC	5.0 mmol/L	(0.9)
LDL	3.1 mmol/L	(0.8)
HDL	1.2 mmol/L	(0.3)
TG	1.6 mmol/L	(1.1)
Total cholesterol*		
<5.2	60.9%	
5.2-6.2	28.8%	
>6.2	9.9%	
LDL*		
<2.6	30.4%	
2.6-3.3	35.9%	
3.4-4.1	23.2%	
4.1-4.9	7.4%	
>4.9	2.1%	
HDL*		
<1.0	16.5%	
1.0-1.5	53.6%	
>1.5	29.5%	
TG*		
<1.7	68.1%	
1.7-2.2	16.4%	
2.3-5.6	14.1%	
>5.6	1.0%	
**Mean eGFR** (ml/min/1.73 m^2^)	84.8	(23.2)
Chronic kidney disease*		
Stage 1	38.5%	
Stage 2	48.8%	
Stage 3	11.7%	
Stage 4	0.3%	
Stage 5	0.1%	
**Mean urine ACR**	10.2 mg/mmol	(42.7)
Proportion normal	67.9%	

TC: total cholesterol; LDL: low density lipoprotein; HDL: high density lipoprotein; TG: triglyceride; ACR: albumin to creatinine ratio.

The article "Prevalence of complications among Chinese diabetic patients in urban primary care clinics: a cross-sectional study" was retracted in 2025. Reason: lack of ethics approval or compliance.

*Percentages may not add up to 100% because of missing data.

In terms of glycaemic control, 51.5% had an HbA1c level of less than 7.0% (Figure 1). 88.4% of patients did not achieve target LDL level (2.6 mmol/L) (Table 2).

**Figure 1:** Distribution of HbA1c values among study population.

15% of patients were on diet control alone (Table 3). 39.1% of them are on both a biguanide and sulphonylurea, while 1.2% are using insulin therapy. Amongst those taking antihypertensives, 36.6% are on monotherapy, 39.3% on dual therapy, and 24.0% are on three or more. Only 20.7% of patients are on statins. In patients with microalbuminuria and macroalbuminuria, 40.7% and 54.5% were on ACEI or ARB respectively.

**Table 3:** Drug use among study population

**Type of therapy**	Proportion of patients*
**Diet alone**	15.0%
**Glucose lowering therapy**	
Metformin	64.5%
Sulphonylurea	54.5%
Glitazone	0.5%
Gliptin	0.1%
Insulin	1.6%
**Anti-hypertensives**	
None	35.4%
ACEI or ARB	38.2%
β-blocker	26.6%
CCB	41.8%
Diuretic	13.2%
**Lipid lowering therapy**	
Statin	22.2%
Fibrate	3.7%
**Aspirin**	9.4%

ACEI: angiotensin converting enzyme inhibitor.

ARB: angiotensin receptor blocker.

CCB: calcium channel blocker.

*Percentages do not add up to 100% because some patients may be taking more than one therapy.

### Prevalence of complications

Table 4 shows the prevalence of complications among our population. Diabetic retinopathy was detected in 12.9% of patients. Nephropathy was present in 38.8%. 67.7% had a urine albumin to creatinine ratio of less than 2.5 mg/mmol and 3.5 mg/mmol among males and females respectively. Neuropathy was present in 2.4%. Overall, 37.9%, 6.7% and 0.3% had single, two and three microvascular complications (among the complications of diabetic retinopathy, nephropathy and neuropathy) respectively (Figure 2). Among male patients, 15% reported to have erectile dysfunction.

**Table 4:** Prevalence of diabetic complications

**Complication**	**Percentage**
**Diabetic retinopathy (n = 1920)**	
Mild non-proliferative	12.1%
Moderate to severe non-proliferative	0.5%
Proliferative	0.3%
**Nephropathy (n = 5986)**	
Incipient	30.9%
Overt	7.9%
**Neuropathy (by monofilament/tuning fork) (n = 386)**	2.4%
Reported numbness	5.4%
Presence of foot ulcer	0.5%
Absent foot pulses	0.2%
Foot deformity	4.3%
Presence of callosity	30.3%
Presence of suspected skin infection	2.2%
Nail abnormalities	7.3%
**Erectile dysfunction (male only)**	15.0%

The article "Prevalence of complications among Chinese diabetic patients in urban primary care clinics: a cross-sectional study" was retracted in 2025. Reason: lack of ethics approval or compliance.

**Figure 2:** Prevalence of complications among study population.

## Discussion

This is the first study looking into the epidemiology of diabetic patients in Hong Kong’s primary care system. The level of diabetic control among our population appears to be comparable with other developed countries [5,6], with around 50% achieving an HbA1c of <7.0%. The majority of patients can be controlled with traditional oral hypoglyaemic agents (OHAs). The much lower use of gliptins and other newer OHAs is mainly because these are self finance items in contrast to traditional medications which are provided without cost, at the time of the study period (the newer drugs are now provided according to the guidelines of the Formulary in Hong Kong). With reference to a previous population study on hypertension-alone patients [7], the pattern of antihypertensive drug usage among our diabetic population is different, with a greater proportion prescribed with an ACEI or ARB. This is likely to be related to coexisting need for renal protection among susceptible patients.

Glycaemic control forms only part of the overall management of diabetes. Despite the well documented evidence on the importance of adequate weight management [8] as well as blood pressure [9,10] and lipid control [11-14], gaps currently still exist as evidenced by the large proportion of patients who are obese, with suboptimal blood pressure control and abnormal lipid levels. That may explain partly the reasons for the relatively high prevalence of incipient and overt nephropathy. Efforts to improve management must be tailored according to the needs of our population, where the majority have a low educational background and a significant proportion being retired and elderly. Increased resources must also be placed in primary care so that drug management can be optimized. Currently although 88.4% have suboptimal lipid levels, only 22.2% are on statin therapy. ACEIs and ARBs are readily available in the clinics reviewed in this study. Although practice guidelines already exist to help doctors in deciding when these are required, further education and reminders must be provided to ensure doctors adhere to evidence-based practice.

Compared with recent primary care literature [15,16], our study population had a lower prevalence of neuropathy (2.4% vs >15% in existing literature) and a higher prevalence of nephropathy (38.8% vs 10.5%). The prevalence of retinopathy was comparable. On the other hand, prevalence studies among hospital-based patients in urban China [17] revealed that our primary care patients had a higher rate of microvascular complications (44.9% vs 34.7%). The reason for these differences in complication prevalence is unclear. However, the detection of neuropathy depends on the use of monofilaments and graduated tuning fork, both of which is user dependent and subject to patient interpretation. We could have missed patients with small-fibre damage. Although we cannot exclude the possibility of underestimating diabetic neuropathy in our program, another cohort of type 2 diabetes patients from seven Asian countries also reported a low prevalence of diabetic neuropathy in Hong Kong (1.9% as compared to the overall prevalence of 15% in seven countries) [18]. Furthermore, our estimate of diabetic neuropathy in Chinese patients is concordant with a recent study in Shanghai reporting a prevalence of peripheral neuropathy of 8.4% in diabetes subjects [19].

The article "Prevalence of complications among Chinese diabetic patients in urban primary care clinics: a cross-sectional study" was retracted in 2025. Reason: lack of ethics approval or compliance.

Despite the low insulin usage rate, good average HbA1c level and short disease duration, our population appears to have a relatively higher prevalence of microvascular complication. Primary care physicians must therefore be aware of this high complication prevalence, educating patients on the importance of early detection irrespective of diabetic control. Recently in England, a form of integrated care, which allowed patients to move seamlessly between primary, community, and secondary care depending on need, and which enhanced interaction, information exchange, and learning across the clinical services was suggested in order to provide high quality diabetes care [20]. Such integration actually requires a good knowledge of the current diabetes care in the different level of settings. Our data would allow a better review of the diabetic patients in primary care to enhance further integration with secondary care.

Limitations of this study include the lack of data on acute complications and the possibility of selection bias, where more patients with worse disease control (including high HbA1c values and those with complications) were recruited into the program, while others with inadequate control or multiple comorbidities have been referred to secondary care. The intention of the program was to include all diabetic patients irrespective of their current disease control status. Nevertheless, further data collection needs to be performed in order to assess whether those who have not yet entered the program are significantly different from this study population. Further studies will also be required in order to see whether our patients with seemingly milder disease will progress at different rates from other populations.

The article "Prevalence of complications among Chinese diabetic patients in urban primary care clinics: a cross-sectional study" was retracted in 2025. Reason: lack of ethics approval or compliance.

## Conclusion

This study aimed to obtain a cross-sectional view of the current level of care among diabetic patients as managed in the primary care setting. Further data collection will be required to assess whether this program will have an impact on diabetic care among our population. More importantly, data from this study demonstrated a high prevalence of microvascular complications among Chinese primary care patients despite achieving adequate HbA1c levels, highlighting the importance of managing all aspects of diabetes including weight, lipid and blood pressure.

## Competing interests

The authors declare that they have no competing interests.

## Authors’ contributions

PKTL/ KK/ AL conceptualised the whole study. KK researched data and wrote the manuscript. KMC, EMTH, ML, SYL and AL reviewed the manuscript. CCS/PKTL contributed to results/discussion and reviewed the manuscript. All authors declare that there are no financial relationships with any organisations that might have an interest in the submitted work, and that no presentations have been made for this research. All authors read and approved the final manuscript.

## Pre-publication history

The pre-publication history for this paper can be accessed here:

http://www.biomedcentral.com/1471-2296/15/8/prepub
